# Jujuboside A Ameliorates Myocardial Apoptosis and Inflammation in Rats with Coronary Heart Disease by Inhibiting PPAR-*α* Signaling Pathway

**DOI:** 10.1155/2022/2285728

**Published:** 2022-06-24

**Authors:** Chunfang Hu, Zhiyuan Zhang, Guixian Song, Li Zhu, Ruzhu Wang, Zhongbao Ruan

**Affiliations:** ^1^Cardiovascular MedicineCardiovascular Medicine, Taizhou People's Hospital, Taizhou 225399, Jiangsu, China; ^2^Dalian Medical University, Dalian 116000, Liaoning, China

## Abstract

**Background:**

Coronary heart disease (CHD) is a chronic disease caused by atherosclerosis (AS), which can cause myocardial ischemia, hypoxia, or necrosis, seriously threatening human health. There is an urgent need for effective treatments and drugs to reduce the various risk factors for coronary heart disease and relieve symptoms of angina pectoris and myocardial infarction in patients. Jujuboside A (JuA) is a triterpenoid saponin extracted from jujube seeds, which has various biological activities such as antioxidant, anti-inflammatory, antiapoptotic, and neuroprotective effects. We study the function of JuA in myocardial injury, dyslipidemia, and inflammation in the CHD rat model, to explore its potential mechanism of improving CHD.

**Methods:**

A rat model of CHD was established by feeding a high-fat diet. The rats were randomly divided into 5 groups (*n* = 6): control group, CHD group, JuA 25 mg/kg group, JuA 50 mg/kg group, and JuA 75 mg/kg group. Echocardiography was used to detect the cardiac function parameters of rats in each group, and then, hematoxylin and eosin staining was used to assess the histopathological injury in myocardial tissues. Levels of blood lipids, myocardial injury indexes, and inflammatory factors of rats in each group were measured by biochemical tests and enzyme linked immunosorbent assay, and the levels of Bax, Bcl-2, c-caspase-3, PPAR-*α*, p65, p-p65, I*κ*B*α,* and p-I*κ*B*α* protein expression in myocardial tissues were detected by western blot.

**Results:**

Compared with the CHD group, JuA therapy significantly improved injury in myocardial tissue and endothelial tissue. It also strengthened cardiac function, while decreasing total cholesterol, triacylglycerol, and low-density lipoprotein cholesterol levels in the serum and increasing high-density lipoprotein cholesterol levels. In addition, JuA also restrained cardiomyocytes apoptosis and inhibited the inflammatory reaction by reducing TNF-*α*, IL-1*β*, and IL-6 expression in myocardial tissues. Furthermore, administration of JuA inhibited the activation of PPAR-*α* pathway by preventing the phosphorylation of p65 and I*κ*B*α* in myocardial tissues of CHD rats.

**Conclusion:**

JuA may improve cardiac function, alleviate myocardial and endothelial injury, and also ameliorate dyslipidemia and inflammatory reaction in rats with CHD, where JuA probably plays a protective role by inhibiting the activation of PPAR-*α* pathway.

## 1. Introduction

Coronary heart disease (CHD), a chronic disease caused by atherosclerosis (AS), is a great threat to human health, which can cause myocardial ischemia, hypoxia, or necrosis [1]. In recent years, with the improvement of people's living standards, the incidence of CHD has been increasing year by year and the age of patients tends to be younger [2]. Studies have shown more than 8.14 million deaths from CHD in 2013, a substantial increase from 5.2 million in 1990 [3–5]. Developing countries have witnessed a more rapid increase in the incidence of CHD. *2021 China Medical Quality Report of Cardiovascular Diseas*es published by National Institute of Hospital Administration (NHC) demonstrated that the incidence of angina pectoris and myocardial infarction reaches 52.7% in hospitalized CHD patients with the mortality of 4.4% [6, 7]. Risk factors for CHD include hypertension, obesity, diabetes, elevated blood cholesterol, smoking, lack of exercise, poor diet, excessive alcohol consumption, and depression [8–11], which aggravate the progression of CHD. Therefore, there is an urgent need for effective therapies and drugs to reduce various risk factors for CHD and relieve angina pectoris and myocardial infarction symptoms in patients.

Peroxisome proliferator-activated receptors (PPARs) are ligand-induced nuclear transcription factors from the nuclear receptor superfamily [12]. PPAR-*α*, an isomer of PPARs, is an important factor in stabilizing the internal environment of lipid metabolism, which can inhibit cyclooxygenase (COX)-2 and activity of monocyte chemoattractant protein (MCP) [13]. Studies have demonstrated that PPAR-*α* plays a key role in regulating lipid metabolism, inflammatory reaction, and endothelial function [14–16]. Meanwhile, PPAR-*α* also has a significant role in CHD. For example, as reported by Shu et al, andrographolide can inhibit endothelial dysfunction and inflammatory reaction in rats with CHD by regulating PPAR-*α* signaling pathway [17]. In addition, activators of PPAR-*α* (fibrates) have been used clinically for the treatment of hyperlipidemia and diabetes for many years [18, 19].

Spine date seed is a dried and mature seed of common jujube from Rhamnaceae, possessing various effects such as arresting sweat, nourishing the liver, and tranquilizing the mind; *Zizyphus jujuba* seed extract has been found to exert multifaceted beneficial pharmacological effects on cardiovascular system including reducing blood lipids, regulating serum lipoproteins, lowering blood pressure, and its antiarrhythmic activity [20, 21]. Jujuboside A (JuA) is a triterpenoid saponin isolated from spine date seed, which has various biological activities such as antioxidative, anti-inflammatory, antiapoptotic, and neuroprotective effects [22–24]. In addition, JuA also has calcium antagonistic and antiatherosclerotic effects, and its mechanism of action is related to its inhibition of excessive proliferation of vascular smooth muscle cells [25]. Several studies have shown that JuA plays an important role in diseases, including Alzheimer's disease [26], lung cancer [27], and diabetes [24]. But there is no report about the role of JuA in CHD. Therefore, this study established a CHD rat model with a high-fat diet to investigate the effects of JuA on cardiac function, myocardial apoptosis, lipid level, and inflammation in CHD rats to preliminarily shed light on its possible mechanism of action.

## 2. Materials and Methods

### 2.1. Establishment of the Animal Model and Intervention

Healthy and SPF-grade SD rats (weighing 200–220 g) aged 6–8 weeks were offered by Nantong University Laboratory Animal Center. All experiments were approved by The Fifth Affiliated Hospital of Nantong University (S20210226-017) Ethics Committee and conducted in accordance with approved guidelines. The CHD rat model was established through methods described in [28]. Briefly, the animals were fed high-fat diet (70% common feed, 10% yolk powder, 10% butter, 7.5% cholesterol, and 2.5% sodium taurocholate) for 8 weeks, and pituitrin 30 U/kg was intraperitoneally injected 24 hours later for 3 consecutive times. Pituitrin can cause coronary artery spasm and vasoconstriction, increase peripheral vascular resistance, and then cause myocardial insufficiency and myocardial injury in rats. The electrocardiogram of the rat was detected, and it showed that the *T* wave was towering, there occurred arrhythmia, and ST segment elevation exceeded 0.1 mV, indicating that the modeling was successful.

Thirty SD rats were randomly divided into five groups (*n* = 6): control group, CHD group, JuA 25 mg/kg group, JuA 50 mg/kg group, and JuA 75 mg/kg group. The rats of control group were fed normal diet for 8 weeks and received intraperitoneal injection of the same amount of distilled water (3 times) and gavage of distilled water (4 weeks). The other rats were fed with high-fat diet to induce CHD. The CHD group was administrated equal volume of distilled water by gastric gavage (4 weeks), while the other groups received JuA at 25 mg/kg/d, 50 mg/kg/d, and 75 mg/kg/d for 4 weeks, respectively [20].

### 2.2. Heart Ultrasound Examination

Twenty-four hours after the last administration, the rats were anesthetized with isoflurane and the chest hair was removed. Rats were fixed in dorsal position, and the cardiac function of the rats in each group was measured by two-dimensional and M-mode echocardiogram. The cross-section graph of parasternal left ventricular long axis was obtained, and the left ventricular ejection fraction (LVEF), left ventricular end-diastolic diameter (LVEDd), left ventricular end-systolic diameter (LVESd), fractional shortening (FS), and other indicators were measured under short-axis *M* ultrasound to evaluate the systolic function of the heart, where FS = (LVEDd − LVESd)/LVEDd [29].

### 2.3. Hematoxylin and Eosin Staining (H&E)

After isolation of rat myocardial tissue, a portion of the tissue was put into formalin solution for fixation before use. As described by Xie et al. [30], the pathological changes of rat myocardium were observed by histological section and HE staining.

### 2.4. Biochemical Tests

Rat myocardial tissues were ground into tissue homogenates with a tissue grinder by adding an appropriate amount of physiological saline. After tissue homogenate or rat serum was centrifuged, the supernatant was taken for spare use. The supernatant was diluted into different concentration gradients of stock solution, and then, an automatic biochemical analyzer was used to investigate the levels of total cholesterol (TC), triglyceride (TG), low-density lipoprotein cholesterol (LDL-C), high-density lipoprotein cholesterol (HDL-C), and endothelin (ET)-1 in rat serum, as well as creatine kinase isoenzyme (CK-MB) and cardiac troponin (cTn) *T* levels in myocardial tissue.

### 2.5. Enzyme-Linked Immunosorbent Assay (ELISA)

Rat myocardial tissue, added with appropriate amount of normal saline, was added into a tissue grinder and ground into tissue homogenates and then centrifuged at 3000 r/min for 10 min at 4°C. The supernatant was taken for testing. The tissue was diluted to the appropriate concentration according to the instructions of the ELISA kit (Wuhan Huamei, China). In brief, the reagents and samples were added to the enzyme label plate in sequence. After the reaction was completed, the absorbance value (OD value) at a wavelength of 450 nm was detected. Finally, according to the standard curve, the levels of tumor necrosis factor-alpha (TNF-*α*) and interleukin-1*β* (IL-1*β*) and IL-6 in myocardial tissue were calculated.

### 2.6. Western Blot (WB)

Total protein was extracted from myocardial tissue of rats in each group by using RIPA lysate, and protein concentration was determined with a BCA kit. Total protein was separated by using 10% SDS-PAGE gels and transferred onto PVDF membranes (Millipore, USA). After being sealed in 5% nonfat dry milk for 2 h, the membranes were incubated overnight at 4°C with primary antibody (Bax, Bcl-2, c-caspase 3, GAPDH, PPAR-*α*, P65, p-P65, I*κ*B*α*, and p-I*κ*B*α*; Abcam, USA). PBST was rinsed for three times, and then, the membrane was probed with secondary antibody (Abcam, USA) for 1 h at room temperature. And then, PBST was washed again and evenly added with the ECL luminescence agent in drops, FliorchemHD2 imaging system was used for scanning analysis and picture acquisition, and protein bands were taken for quantitative analysis by using Image J software.

### 2.7. Statistical Analysis

All result data were expressed as means ± standard deviation (SD) and plotted with Graphpad Prism 9. SPSS 21.0 software was used for statistical analysis. One-way ANOVA was used for comparison among groups. There were significant differences in one-way ANOVA. When the variance was homogeneous, LSD test was used for comparison among multiple groups. *P* < 0.05 indicated significant difference.

## 3. Results

### 3.1. JuA Improved Cardiac Function and Alleviated Myocardial Injury in Rats with CHD

We evaluated the cardiac function and myocardial histopathological damage in rats of each group using echocardiography and HE staining. The results showed that LVEF and FS were significantly decreased, while LVEDd and LVESd were significantly increased in the CHD group compared with the control group (*P* < 0.01); JuA therapy could significantly raise LVEF and FS in CHD rats (*P* < 0.05) and greatly reduce LVEDd and LVESd (*P* < 0.05) depending on concentration (Figures 1(a)–1(d)). The images of HE staining depicted normal myocardial morphology, clear cell boundary, and an orderly arrangement in the control group. The CHD group appeared to have swollen myocardial cells, disorganized myocardial fibers, necrosis, and atrophy of myocardial cells; however, these symptoms were greatly alleviated with JuA treatment, and the improvement effects became more obvious with increasing concentration (Figure 1(e)). These results indicate that JuA could improve cardiac function and attenuate myocardial injury in CHD rats in a concentration-dependent manner.

### 3.2. JuA Reduced Blood Lipid Levels in CHD Rats

Dyslipidemia is a high risk factor for coronary heart disease [31]. TC, TG, and LDL-C and HDL-C are the main components of plasma lipids and play a key role in the development of coronary heart disease [13]. Biochemical tests were used to measure TC, TG, LDL-C, and HDL-C levels in plasma. The results showed that compared with the control group, the serum levels of TC, TG, and LDL-C in the CHD group were significantly increased (*P* < 0.01), while the level of HDL-C was significantly decreased (*P* < 0.001); administration of JuA reduced the levels of serum TC, TG, and LDL-C in CHD rats and increased the level of HDL-C (*P* < 0.01) in a dosage-dependent manner (Figures 2(a)–2(d)). Collectively, JuA may improve the risky lipid environment in CHD rats and higher concentrations of JuA could have a larger improvement effect.

### 3.3. JuA Inhibited Apoptosis of Cardiomyocytes in CHD Rats

Bcl-2 and Bax are representatives of antiapoptotic and proapoptotic proteins in the Bcl-2 family [32], and Caspase-3 is the executor of apoptosis [33]. To further investigate the effect of JuA on myocardial apoptosis in CHD rats, we checked up the expression levels of Bcl-2, Bax, and c-caspase-3 in myocardial tissue of CHD rats. As revealed by WB, CHD rats had decreased expression of Bcl-2 protein and increased protein expression of Bax and c-caspase-3 in the myocardial tissue (*P* < 0.01). After JuA therapy, the expression of Bcl-2 in the myocardial tissue of CHD rats significantly rose and Bax and c-caspase-3 significantly declined (*P* < 0.01) in a concentration-dependent manner (Figures 3(a)and 3(b)). This means that JuA could inhibit the myocardial cells apoptosis in CHD, and its antiapoptotic effect may be more significant at high concentrations.

### 3.4. JuA Alleviated Myocardial Injury and Endothelial Injury in CHD Rats

cTnT, CK-MB, and ET-1 are commonly used markers of myocardial injury and endothelial injury, as they may reflect the presence and extent of myocardial and endothelial injury [34, 35]. Therefore, we measured the levels of serum CK-MB, cTnT, and ET-1 by ELISA to evaluate the effects of JuA on myocardial and endothelial injury in CHD rats. As shown in Figures 4(a)–4(c), with serum CK-MB, cTnT, and ET-1 in the CHD group significantly higher than those in control group (*P* < 0.001), JuA dose-dependently reduced their levels in the serum (*P* < 0.05). These results confirm that JuA treatment could alleviate myocardial and endothelial injury in CHD rats.

### 3.5. JuA Inhibited the Inflammatory Reaction in Rats with CHD

Inflammatory reaction is crucial to the development of CHD [36]. To comprehensively explore the effect of JuA on the inflammatory reaction in CHD rats, we measured the levels of proinflammatory factors (TNF-*α*, IL-1*β*, and IL-6) in rats of each group. ELISA results showed that the levels of TNF-*α*, IL-1*β*, and IL-6 in the myocardial tissue of CHD rats were significantly increased compared with the control group (*P* < 0.001); the levels of TNF-*α*, IL-1*β*, and IL-6 in the myocardial tissue of JuA group were significantly lower than those in the CHD group (*P* < 0.05) in a concentration-dependent manner (Figures 5(a)–5(c)). In summary, JuA could reduce myocardial inflammatory reaction in CHD rats.

### 3.6. JuA Inhibited Activation of PPAR-*α* Signaling Pathway in CHD Rats

Finally, in order to verify whether PPAR-*α* signaling pathway is related to the protective effect of JuA in CHD, we investigated the expression levels of PPAR-*α* signaling pathway-related proteins in rats of each group. Using WB, we found downregulation of PPAR-*α* in the myocardial tissues of rats in the CHD group relative to the control group (*P* < 0.01) and upregulation of p-p65 and p-I*κ*B*α* (*P* < 0.01). However, their expressions were restored greatly in the presence of JuA, as demonstrated by an increase in PPAR-*α* expression and a decrease in p-p65 and p-I*κ*B*α* (*P* < 0.01) in a concentration-dependent manner (Figures 6(a) and 6(b)), which indicates that JuA could inhibit the activation of PPAR-*α* pathway in CHD rats.

## 4. Discussion

CHD is a disease of myocardial ischemia, hypoxia, and injury, caused by vascular lumen occlusion or endothelial damage due to atherosclerotic lesions in the coronary vessels, whilst myocardial ischemia could lead to oxygen supply deficiency and myocardial apoptosis affecting cardiac function [37]. Besides, acute ischemia of the myocardium induces injury, increased permeability of cellular membrane, and increased levels of serum CK-MB and cTnT [38–40]. ET-1 is a potent vasoconstrictor released by endothelial cells, and serum ET-1 levels could be used as a diagnostic indicator of endothelial injury [41, 42]. Apoptosis could occur in the myocardium when in cases of ischemia and injury [40]. In this study, we found that LVEF and FS were significantly decreased, while LVEDd and LVESd increased in CHD rats with disorganized myocardial fibers and necrosis and atrophy of myocardial cells. Meanwhile, the CHD rats exhibited increased levels of CK-MB, cTnT, and ET-1 and cell apoptosis level. The above phenomena suggested that the cardiac function, myocardial tissue, myocardial cells, and endothelial cells of CHD rats were damaged, consistent with the results of previous research on CHD myocardial injury [17, 40]. Importantly, after we administrated JuA to the CHD rats, the symptoms described above were alleviated. LVEF and FS were significantly increased, LVEDd and LVESd decreased, and CK-MB, cTnT, and ET-1 levels decreased. The degree of myocardial injury was alleviated, and myocardial apoptosis was inhibited, which suggested that JuA could improve cardiac function, attenuate myocardial injury and vascular endothelial injury, and inhibit myocardial apoptosis in CHD rats. Consistently, Wang and Han et al. also concluded that JuA inhibited apoptosis, improved cell viability, and protected cardiomyocytes from damage in H9c2 [22, 43].

At present, dyslipidemia has been widely recognized in the pathogenesis of CHD and it is related to low levels of HDL and high levels of TG, TC, and LDL, especially high LDL levels, which is involved in the etiology of coronary atherosclerosis [44, 45]. The study actually depicted that the levels of serum TG, TC, and LDL were significantly increased in CHD rats, while HDL declined, indicating successful establishment of a CHD rat model through high-fat diet, which laid the foundation for the subsequent study about JuA function. Of note, JuA treatment significantly reduced the levels of serum TC, TG, and LDL-C and restored the level of HDL-C in CHD rats. These alterations indicate that JuA may reduce blood lipid and ameliorate dyslipidemia in CHD, which was consistent with the finding by Wu Yulan that spine date seed could pharmacologically lower blood lipids [21].

Afterwards, studies have reported that the inflammatory reaction plays an important role in the progress of CHD and that neutrophils, monocytes, macrophages, and lymphocytes induced by the inflammatory reaction contributes to CHD development [41], as increased expression of inflammatory factors aggravates the progression of CHD [46]. A significant decline in the levels of TNF-*α*, IL-1*β,* and IL-6 was also found in the myocardial tissue of CHD rats in the present study. And, their levels were significantly reduced after JuA treatment, suggesting anti-inflammatory activity of JuA. Wang's study also noted that JuA was able to reduce the levels of IL-1*β* and TNF-*α* in the small intestinal tissue [24].

PPAR-*α* is mainly expressed in the heart, liver, kidney, and other tissues, and it may inhibit NF-*κ*B-mediated pathways and reduce the secretion of proinflammatory factors and lessen PPAR-*α* expression in ischemic myocardial tissue [47]. The PPAR-*α* signaling pathway was not only associated with endothelial dysfunction and inflammatory reaction in CHD rats [17], but also with lipid metabolism [48]. In this study, we found that PPAR-*α* signaling pathway was significantly activated in the myocardial tissue of CHD rats and administration of JuA greatly inhibited the phosphorylation of p65 and I*κ*B*α* in the myocardial tissue of CHD rats, suggesting that JuA could inhibit activation of PPAR-*α* signaling pathway, which was compatible with results in the study by Shu et al. [17].

This study also has limitations. Although JuA was found to inhibit PPAR-*α* pathway by WB, whether JuA exerts its protective effects on anti-inflammation, antiapoptosis, and lipid regulation in CHD rats through this pathway was not further verified in experiments. Moreover, it has been proved in this study that JuA could protect cardiomyocytes through MAPK, AKT, and PI3K/Akt/mTOR signaling pathways [22, 43]. Therefore, the specific mechanisms underlying JuA functions in CHD require further investigation and experiment.

## 5. Conclusions

Collectively, JuA can not only improve cardiac function, ameliorate myocardial injury and endothelial injury, and inhibit apoptosis of myocardial cells in CHD rats but also improve blood lipid levels, in addition to reducing the inflammatory response, in a concentration-dependent manner. The role of JuA in CHD may be associated with its inhibition of activation of the PPAR-*α* pathway.

## Figures and Tables

**Figure 1:** Effect of JuA on cardiac function and myocardial injury in CHD rats. (a–d) LVEF, LVEDd, LVESd, and FS were measured by echocardiography; (e) HE staining was used to observe the pathological injury level of myocardium in each group (100x and 400x times). ^###^*P* < 0.001 vs. control group; ^*∗*^*P* < 0.01, ^*∗∗*^*P* < 0.01, and ^*∗∗*^*P* < 0.001 vs. CHD group.

**Figure 2:** Effect of JuA on lipid levels in CHD rats. The serum levels of TC (a), TG (b), LDL-C (c), and HDL-C (d) in each group of rats were detected in biochemical tests. ^###^*P* < 0.001 vs. control group; ^*∗*^*P* < 0.01, ^*∗∗*^*P* < 0.01, and ^*∗∗*^*P* < 0.001 vs. CHD group.

**Figure 3:** Effect of JuA on cardiomyocyte apoptosis in CHD rats. (a) WB was used to detect the protein expression levels of Bax, Bcl-2, and c-caspase-3 in the myocardial tissues of rats in each group; (b) Image J was used to analyze the relative protein expression levels of Bax, Bcl-2, and c-caspase-3. ^###^*P* < 0.001 vs. control group; ^*∗*^*P* < 0.01, ^*∗∗*^*P* < 0.01, and ^*∗∗*^*P* < 0.001 vs. CHD group.

**Figure 4:** Effect of JuA on myocardial injury and endothelial injury in CHD rats. Biochemical tests of CK-MB (a) and cTnT (b) levels in myocardial tissue of rats in each group; (c) biochemical tests of ET-1 levels in the serum of rats in each group. ^###^*P* < 0.001 vs. control group; ^*∗*^*P* < 0.01, ^*∗∗*^*P* < 0.01, and ^*∗∗*^*P* < 0.001 vs. CHD group.

**Figure 5:** Effect of JuA on inflammation in CHD rats. The levels of TNF-*α* (a), IL-1*β* (b), and IL-6 (c) in the myocardial tissue of rats in each group were detected by ELISA. ^###^*P* < 0.001 vs. control group; ^*∗*^*P* < 0.01, ^*∗∗*^*P* < 0.01, and ^*∗∗*^*P* < 0.001 vs. CHD group.

**Figure 6:** Effect of JuA on PPAR-*α* signaling pathway in CHD rats. (a) WB was used to detect the protein expression levels of PPAR-*α*, p65, p-p65, I*κ*B*α*, and p-I*κ*B*α* in cardiomyocytes of rats in each group; (b) Image J was used to analyze the protein expression levels of PPAR-*α* and the ratios of p-p65/*p*65 and p-I*κ*B*α*/I*κ*B*α*. ^###^*P* < 0.001 vs. control group; ^*∗*^*P* < 0.01, ^*∗∗*^*P* < 0.01, and ^*∗∗*^*P* < 0.001 vs. CHD group.

## Data Availability

The data used to support the findings of this study are available from the corresponding author upon request.
